RETRACTED

# miR-381 Regulates Neural Stem Cell Proliferation and Differentiation via Regulating Hes1 Expression

**DOI:** 10.1371/journal.pone.0138973

**Published:** 2015-10-02

**Authors:** Xiaodong Shi, Chunhua Yan, Baoquan Liu, Chunxiao Yang, Xuedan Nie, Xiaokun Wang, Jiaolin Zheng, Yue Wang, Yulan Zhu

**Affiliations:** 1 Department of Neurology, The Second Affiliated Hospital of Harbin Medical University, Harbin, 150081, PR China; 2 Department of Respiratory, The Second Affiliated Hospital of Harbin Medical University, Harbin, 150081, PR China; 3 Department of anatomy, Harbin Medical University, Harbin, 150081, PR China; 4 Department of Occupational Health, College of Public Health, Harbin Medical University, Harbin, 150081, PR China; Peking Union Medical College Hospital, CHINA

## Abstract

Neural stem cells are self-renewing, multipotent and undifferentiated precursors that retain the capacity for differentiation into both glial (astrocytes and oligodendrocytes) and neuronal lineages. Neural stem cells offer cell-based therapies for neurological disorders such as Alzheimer's disease, Parkinson's disease, Huntington's disease and spinal cord injuries. However, their cellular behavior is poorly understood. MicroRNAs (miRNAs) are a class of small noncoding RNAs involved in cell development, proliferation and differentiation through regulating gene expression at post-transcriptional level. The role of miR–381 in the development of neural stem cells remains unknown. In this study, we showed that overexpression of miR–381 promoted neural stem cells proliferation. It induced the neural stem cells differentiation to neurons and inhibited their differentiation to astrocytes. Furthermore, we identified HES1 as a direct target of miR–381 in neural stem cells. Moreover, re-expression of HES1 impaired miR-381-induced promotion of neural stem cells proliferation and induce neural stem cells differentiation to neurons. In conclusion, miR–381 played important role in neural stem cells proliferation and differentiation.

## Introduction

Neural stem cells are undifferentiated precursors, self-renewing cell populations that retain the ability to differentiate to both glial (astrocytes and oligodendrocytes)and neuronal lineages[1–5]. Neural stem cells are found in the adult and developing mammalianCNS (central nervous system)[6, 7]. Recent data show that neural stem cells can serve as cell replacement therapies for neurological disorders such as Alzheimer's disease, Parkinson's disease, Huntington's disease and spinal cord injuries[8–11]. Despite the great hope of using neural stem cells for clinically intervention, it is still a long distance before clinical application of neural stem cells[12–14]. Therefore, it is urgent to understand the molecular pathways controlling NSC proliferation and differentiation.

RETRACTED

MicroRNAs (miRNAs) are a group of naturally occurring, conserved small non-coding, ~22-nucleotide RNA molecules that can inhibit translation or transcription by targeting protein-coding genes[15–19]. miRNAs are involved in a lot of biological functions such as cellular development, differentiation, proliferation, andapoptosis[20–23]. Deregulation of miRNAs has been found in various tumors including gastric cancer, laryngeal cancer, hepatocellular carcinoma, glioblastoma and ovarian carcinoma[16, 24–28]. Recently studies also found that miRNAs played an important role in stem cell fate determination and self-renewal by controlling the expression of stem cell regulators[3, 29–31].

In this study, we demonstrated that overexpression of miR–381 promoted neural stem cells proliferation and differentiation to neurons while it inhibited their differentiation to astrocytes. Furthermore, we identified Hairy and enhancer of split 1 (Hes1) as a direct target of miR–381 in neural stem cells.

## Materials and Methods

### Ethics Statement

This study was approved by the ethical board of the institute of The Second Affiliated Hospital of Harbin Medical University and complied with Declaration of Helsinki.

### Cell Culture and Transfection

Rats were sacrificed by CO2 asphyxiation and neural stem cells were isolated from 13.5 days embryos of Wistar rats and cultured in growth medium with the 1% N2 (Gibco), 10 ng/ml bFGF (R&D), and 20 ng/ml human EGF (R&D) supplement. Primary neurospheres were digested using 0.25% trypsin to derive clone neurospheres. miR–381 mimic and scramble were purchased from Ambion. The transfection of miR–381 mimics and scramble (20ng/ml), Hes–1 vector and related controls was performed using Lipofectamine 2000 (Invitrogen) following to the manufacturer’s instruction.

### Immunocytochemistry

Cells were fixed with paraformaldehyde (4%) and then permeabilized by using 0.2% Triton-X. After blocking with goat serum (10%), cells were incubated with primary antibodies nestin (R&D, Minneapolis, MN, MAB1259), at 4°C overnight and then incubated the fluorescence labeled secondary antibodies. Nuclei were counter stained with DAPI (Vector labs, Burlingame, CA, H1200).

### Cell Proliferation

Cell proliferation was measured by using the Counting kit 8 (CCK8) assay (Dojindo, Kumamoto, Japan) following to the manufacturer’s information. Proliferation rates were evaluated at 0, 24, 48 and 72 h after treatment. The OD (optical density) was evaluated at a wavelength of 450 nm.

### qRT-PCR

Total RNA was isolated from the cells using Trizol reagent (Invitrogen, Carlsbad, CA, USA). Real-time PCR was done to detect the expression of miRNA and mRNA using SYBR Green PCR Kit (QIAGEN) on 7500 Real-Time PCR System (Applied Biosystems).The PCR(polymerase chain reaction) was performed at 95°C for 8 min, then followed by 42 cycles at95°C for 10 s, 60°C for 40 s, and 72°C for 1 s. The primer for Hes1 forward primer 5’-TGAAGGATTCCAAAAATAAAATTCTCTGGG–3’ and reverse primer 5’-CGCCTCTTCTCCATGATAGGCTTTGATGAC–3’; β-tubulin III forward primer 5’-AGCAAGGTGCGTGAGGAGTA–3' and reverse primer 5’-AAGCCGGGCATGAAGAAGT–3’; Nestin forward primer 5’- GATCTAAACAGGAAGGAAATCCAGG–3’ and reverse primer 5’- TCTAGTGTCTCATGGCTCTGGTTTT–3’; GFAP forward primer 5’-CAACGTTAAGCTAGCCCTGGACAT–3’, and reverse primer: 5’-CTCACCATCCCGCATCTCCACAGT–3’ and GAPDH was forward primer 5’-ATTCCATGGCACCGTCAAGGCTGA–3’, reverse primer 5’-TTCTCCATGGTGGTGAAGACGCCA–3’.

RETRACTED

### Western Blot

Proteins were isolated from cells and then and separated on 12% SDS-PAGE gel. Then, it was transferred to PVDF membranes (Amersham, Buckinghamshire, UK). The membrane was blocked with milk (5%) and incubated with primary antibody as following: Nestin, β-tubulin III, GFAP, Hes1 and GDPDH (Sigma) for 2 hours. The blot was probed with HRP-conjugated secondary antibodies for 1 hour. The signal was evaluated by ECL kit(Millipore, MA, USA).

### Luciferase Reporter Assay

The WT (wide type) or MT (mutant) 3’UTR of HES1 was amplified using PCR and cloned to the pGL3-luciferase reporter plasmid (Promega, Madison, WI, USA). Cell was transfected with miR–381 or scramble and luciferase reporter plasmid and the Renilla luciferase (Promega, Madison, WI, USA) using Lipofectamine 2000 (Invitrogen). Luciferase activity was performed using the Dual-Luciferase Reporter reagent (Promega) following to the manufacturer’s information.

### Statistical Analysis

All data were shown as means ± SD. The difference between two groups was used Student’s t test or One-way ANOVA was performed to analyze the more than two groups.

## Results

Neural stem cells could proliferate and differentiate into neurons and astrocytes Isolated cells proliferated and formed neurospheres on the second day after isolation (Fig 1A). These neurospheres also expressed the NSC-specific marker nestin (Fig 1B). Three days after withdraw of bFGF, these neurospheres differentiated into neurons and astrocytes (Fig 1C and 1D), thus confirming the identity of isolated cells as Neural stem cells.

**Fig 1:** Neural stem cells could proliferate and differentiate into neurons and astrocytes. (A) Representative photomicrograph of neurospheres in culture. (B) Immunocytochemical staining of purified NSCs with Nestin. (C) Immunocytochemical staining of purified protoplasmic astrocytes with GFAP. (D) Immunocytochemical staining of purified neurons with β-tubulin-III. (E) Nucleus staining of differentiated cells from NSCs with DAPI.

RETRACTED

### miR–381 Promoted Neural Stem Cells Proliferation

We confirmed that miR–381 mimics could promote the expression of miR–381 in neural stem cells (Fig 2A). CCK–8 analysis demonstrated that overexpression of miR–381 increased neural stem cells proliferation (Fig 2B). In addition, miR–381 overexpression promoted the mRNA and protein expression of nestin (Fig 2C and 2D).

**Fig 2:** miR–381 promoted neural stem cells proliferation. (A) The expression of miR–381 was measured by qRT-PCR. (B) CCK–8 was performed to detect the neural stem cells proliferation. (C) The mRNA expression of nestin was detected by qRT-PCR. (D) The protein expression of nestin was measured by Western blot. **p<0.01 and ***p<0.001.

### miR–381 Promoted Neural Stem Cells Differentiation to Neurons

miR–381 promoted neural stem cells differentiation to neurons as confirmed by immunofluorescence (Fig 3A). miR–381 overexpression promoted the mRNA and protein expression of β-tubulin III (Fig 3B and 3C).

**Fig 3:** miR–381 promoted neural stem cells differentiation to neurons. (A) Immunocytochemical staining of purified neurons with β-tubulin-III. (B) The mRNA expression of β-tubulin-III was detected by qRT-PCR. (C) The protein expression of β-tubulin-III was measured by Western blot.***p<0.001.

### miR–381 Inhibited Neural Stem Cells Differentiation to Astrocytes

miR–381 inhibited neural stem cells differentiation to astrocytesas confirmed by immunofluorescence (Fig 4A). miR–381 overexpression repressed the mRNA and protein expression of GFAP (Fig 4B and 4C).

**Fig 4:** miR–381 inhibited neural stem cells differentiation to astrocytes. (A) Immunocytochemical staining of purified protoplasmic astrocytes with GFAP. (B) The mRNA expression of GFAP was detected by qRT-PCR. (C) The protein expression of GFAP was measured by Western blot.***p<0.001.

### Hes1 Was the Direct Target of miR–381 in Neural Stem Cells

Hes1 was predicted to be target gene ofmiR–381 by TargetScan (Fig 5A).As shown in Fig 5B,miR-381repressed the luciferase activity of wild type 3’UTRof Hes1vector compared to that mutant 3’UTR of Hes1 vector (Fig 5B). Overexpression of miR–381 inhibited HES1 protein expression (Fig 5C).

**Fig 5:** Hes1 was the direct target of miR–381 in neural stem cells. (A) Hes1 was predicted to be target gene ofmiR–381 by TargetScan. (B) Luciferase reporter assay was done to confirm the predictions in neural stem cells. (C) The protein expression of Hes1 was measured by Western blot in neural stem cells.***p<0.001.

RETRACTED

### miR–381 Promoted Neural Stem Cells Proliferation and Differentiation to Neurons by Targeting Hes1

We confirmed thatHes1 vector can promote the expression of Hes1 in neural stem cells (Fig 6A). Overexpression of Hes1 can impair miR-381-induced promotion of neural stem cells proliferation (Fig 6B). Ectopic expression of Hes1 inhibited miR-381-induced nestin mRNA and protein expression in neural stem cells (Fig 6C and 6D). Hes1 overexpression can repress miR-381-induced β-tubulin III mRNA and protein expression in neural stem cells (Fig 6E and 6F). Hes1 overexpression can promoted miR-381-inhibited GFAP mRNA and protein expression in neural stem cells (Fig 6G and 6H).

**Fig 6:** miR–381 promoted neural stem cells proliferation and differentiation to neurons by targeting Hes1. (A) The protein expression of Hes1 was measured by Western blot in neural stem cells. (B) CCK–8 was performed to detect the neural stem cells proliferation. (C) The mRNA expression of Hes1 was measured by qRT-PCR in neural stem cells. (D) The protein expression of Hes1 was measured by Western blot in neural stem cells. (E) The mRNA expression of β-tubulin-III was measured by qRT-PCR in neural stem cells. (F)The protein expression of β-tubulin-III was measured by Western blot in neural stem cells. (G) The mRNA expression of GFAP was measured by qRT-PCR in neural stem cells. (F)The protein expression of GFAP was measured by Western blot in neural stem cells.**p<0.01 and ***p<0.001.

## Discussion

In this study, we demonstrated that overexpression of miR–381 promoted neural stem cells proliferation and differentiation to neurons while it inhibited the neural stem cells differentiation to astrocytes. Furthermore, we identified HES1 as a direct target of miR–381 in neural stem cells. Moreover, re-expression of HES1 impaired miR-381-induced promotion of neural stem cells proliferation and induce neural stem cells differentiation to neurons. Therefore, it is implicated that miR–381 plays important role in neural stem cells proliferation and differentiation.

Previous studies showed that miR–381 acted an important role in biological functions in both noncancerous and cancerous conditions[32–34]. For example, Lee et al[35]. found that miR–381 overexpression inhibited the capacity of colony-forming of malignant mast andnormal cell lines. Another study also found that miR–381 repressed the renal cancer cells proliferation[36]. Moreover, Zhou et al[37]. revealed that miR–381 repressed cell migration and proliferation esophageal squamous cell carcinoma (ESCC). In addition, Hou et al[34]. found that miR–381 expression was upregulated in arthritic cartilage and during chondrogenesis. miR–381 may contribute to absorption of the cartilage matrix by inducing MMP–13 and repressing type II collagen. However, the role of miR–381 in neural stem cells was unknown. In our study, we showed that overexpression of miR–381 promoted neural stem cells proliferation and differentiation to neurons while it inhibited the neural stem cells differentiation to astrocytes.

RETRACTED

Hes genes are mammalian homologues of Enhancer of split and Drosophila hairy that encode bHLH (basic helix-loop-helix) transcriptional repressors[38–40]. Hes1 is a downstream target of Notch signaling and it is highly expressed in the central nervous system[41, 42]. Previous studies demonstrated that Hes1 played an important role in the development of central nervous system[43–45]. Hes1 was considered as crucial in repressing neuronal differentiation[41].The expression ofHes1 was essential for the maintenance of neural stem cells in the embryonic brain; however, overexpression of Hes1 repressed the differentiation and proliferation of neural stem cells[46–48]. Moreover, downregulation of Hes1 induced neural stem cells differentiation into mature neurons[49]. Furthermore, knockdown of Hes1 increased neuronal differentiation through upregulatingMash–1 (the neural differentiation factor)[50].Tan et al. reported that miR–9 could promote the neural stem cells proliferation and differentiation to neurons by regulating Hes1 expression indeveloping brain[4].However, the underlying mechanisms of these are still unclear. Our study demonstrated that the ability of miR–381 to inhibit Hes1 expression might provide one such mechanism of post-transcriptional regulation of Hes1. In our study, we found that Hes1 as a direct target gene of miR–381 in neural stem cells. Firstly, the complementary sequence ofHes1 was predicted to be target gene ofmiR–381. Secondly, the data of luciferase reporter assay proved that miR–381 repressed the luciferase activity of wild type 3’UTR of HES1 vector compared to that mutant 3’UTR of HES1 vector. Thirdly, overexpression of miR–381 inhibited Hes1 protein expression in neural stem cells. The role of Hes1 was further supported by the results that promotion in neural stem cells proliferation and differentiation into neurons was attenuated by re-introduction of Hes1.These data indicate that miR-381play an important role in the proliferation and differentiation of neural stem cells at least partly mediated by inhibiting Hes1 expression in neural stem cells development.

In conclusion, our data demonstrated an important role of miR–381 in the regulation of proliferation, differentiation of neural stem cells. Our study also showed that miR–381 mediated the proliferation and differentiation of neural stem cells by regulating the Hes1 expression.
